# E-Commerce Picture Text Recognition Information System Based on Deep Learning

**DOI:** 10.1155/2022/9474245

**Published:** 2022-01-03

**Authors:** Bin Zhao, WenYing Li, Qian Guo, RongRong Song

**Affiliations:** ^1^School of Economics and Management, Bengbu University, Bengbu, Anhui 233030, China; ^2^Anhui Radio and Television University, Hefei Branch, Hefei, Anhui 230001, China

## Abstract

For the accuracy requirements of commodity image detection and classification, the FPN network is improved by DPFM ablation and RFM, so as to improve the detection accuracy of commodities by the network. At the same time, in view of the narrowing of channels in the application of traditional MWI-DenseNet network, a new GTNet network is proposed to improve the classification accuracy of commodities.The results show that at different levels of evaluation indexes, the dpFPN-Netv2 algorithm improved by DPFM + RFM fusion has higher target detection accuracy than RetinaNet-50 algorithm and other algorithms. And the detection time is 52 ms, which is significantly lower than 90 ms required for RetinaNet-50 detection. In terms of target recognition, compared with the traditional MWI-DenseNet neural network, the computation amount of the improved MWI DenseNet neural network is significantly reduced under different shunt ratios, and the recognition accuracy is significantly improved. The innovation of this study lies in improving the algorithm from the perspective of target detection and recognition, so as to change the previous improvement that only can be made in a single way.

## 1. Introduction

With the maturing of artificial intelligence and image processing technology, the unmanned sales are changing the Commodity sales model. It can be seen that the image detection and classification methods are widely used as an important technical support for unmanned sales. Among them, the target detection can be divided into two-stage detection method based on target region and end-to-end one-stage detection method [1, 2]. Where, the detection methods based on target region include Faster-RCNN [3], etc., and the end-to-end detection methods include You Only Live Once (YOLO), Single Shot MultiBox Detector(SSD),RetinaNet,etc. [4–8]. Segmentation model can be divided into semantic segmentation and instance segmentation. Here, the semantic segmentation models include SegNet, etc. [9–11], and the instance segmentation models include Mask-RCNN, etc. [12, 13]. With the wide application of deep learning, on the basis of target detection, the neural networks such as Convolutional Neural Networks, VGGNet, etc., are applied to classification. But in the application of neural networks, increasing the network layers and amplifying the channels in the network feature graph, the effect of “widening and deepening” of convolutional neural network can be realized. Although it can greatly improve the network performance, it is at the cost of increasing the parameters and increasing the computations. This makes network deployment difficult and reduces the timeliness of network applications.In the context of network lightweight, MWI-DenseNet can repeatedly reference the feature maps by virtue of the built-in multipath dense connection mechanism. Thus, it greatly reduces the computations and parameters. And on the premise of ensuring classification accuracy, it greatly improves network efficiency and network adaptability. The dense connection mechanism has the advantage of feature reuse, but it also causes different layers to repeatedly reference the gradient information of the same layer for parameter optimization, which results in poor optimization effect of network learning.The network update relies heavily on the deep gradient information. But under the dense connection mechanism, the deep gradient information mainly comes from the shallow repeated gradient information. This will inevitably affect the deep learning ability. In this regard, CSPNet further enriches the gradient propagation path by crossing the stage path to avoid the repeated reference of the same gradient information [14].

Inspired by this, this paper uses the deep gradient flow truncation strategy to improve the multipath integration dense connection block and transition layer structure, thus creating a new gradient truncation convolutional network (GTNet). It has obvious advantages, such as less computation, high classification accuracy, large gradient difference, and so on.

## 2. Commodity Inspection Based on FPN

The fusion feature pyramid convolution network constructed in this paper takes DenseNet as the backbone network. It defines the feature graph of some layers of DenseNet as the original feature pyramid [15–18].Then the DPFM module is used to implement the fusion of the three layer feature maps, which are a certain feature diagram, the front and rear layer feature diagram in the original feature pyramid. Under the participation of more DPFM modules, each predict layer gets enough semantic information and precise location information, which can accurately identify objects of all sizes.

In addition, the process reuse feature diagram shows that the calculation amount of feature fusion is greatly reduced. And the efficiency of target detection is improved effectively. First of all, the DPFM module is used to build FPN-Net vl. Then, the RFM module is used to carry on the feature fusion of FPN-Net vl. Finally, the dual-path fusion feature pyramid convolution network FPN-Net v2 was constructed. The above process is shown in Figure 1.

### 2.1. Dual-Path Feature Fusion Module

Figure 2 shows the structure of the DPFM module.

The traditional feature fusion module FPN only has a top-down fusion path. So it can only realize the feature fusion between the previous layer and the current layer. Due to the low reuse rate of feature layer, the fusion of multiple layer is required, which can increase the amount of computation. What's more, it is difficult to fully retain the location information. Different from FPN module, the DPFM module realizes feature fusion of previous layer (*i*+1) − *thlayer* and current layer (*i* − 1) − *thlayer* through top-down fusion path. And it can carry out the feature fusion of latter layer (*i* − 1) − *thlayer* and current layer (*i* − 1) − *thlayer* through bottom-up fusion [19].

The multiple layer feature diagrams are fused by multiple DPFM loops, which makes DPFM + RFM fusion feature pyramid detection network formed. It is shown as Figure 3.

Figure 3 shows the two fusion. Where, the red line represents the top-down fusion path, and the blue line represents the bottom-up fusion path. Specifically, in the red line, the feature graph of previous layer (*i*+1) − th is input. After 1 × 1 convolution, the number of output channels is consistent with the feature graph of current layer (*i*) − *th*. Then, the bilinear interpolation algorithm is introduced to perform Upsample and (*i*+1) fusion input is obtained. In the blue line, the feature graph of later layer (*i* − 1) − *th* is input. After 1 × 1 convolution, the number of output channels is consistent with the feature graph of current layer (*i*) − *th*. Then, the pass though algorithm is introduced to perform Downsample and (*i* − 1) fusion input is obtained. After that, (*i* − 1) fusion input (*i* − 1) − *th* and (*i*) − *th* are spliced in the channel dimension. The spliced feature graph is performed with 3 × 3 convolution, and the final fusion feature layer can be obtained. The number of size channel is consistent with (*i*) − *th* [20–23].

In Figure 3, the DPFM module corresponding to the 4-th layer fuses the front 3-th layer, the current 4-th layer and the rear 5-th layer. The fusion result is used as the input of the top-down fusion path of the DPFM module corresponding to the 3-th layer. At the same time, the 2-th layer is used as the input of the bottom-up fusion path of the DPFM module corresponding to the 3-th layer, and the fusion feature operation is repeated. The multiplex fusion feature mechanism shown in the aforementioned process greatly expands the position information and semantic information of the prediction layer. The fewer original feature layer in the built-in Back Bone not only facilitates module deployment but also reduces the amount of computation. The bidirectional fusion of deep and shallow information is repeated. First of all, it can alleviate the problem of feature information loss caused by pooling. Then, the rich semantic information and accurate location information to the prediction layer can be provided. Finally, the target detection can be precisely achieved. From the application effect, the detection accuracy of cyclic multiplexing bidirectional feature fusion pyramid network is relatively ideal. Especially, it can accurately detect small size objects, and it requires less parameter amount and calculation amount. Thus, the detection efficiency can be improved.

### 2.2. Recombination and Fusion Module

After introducing the recombination and fusion module, the semantic characterization capability of feature pyramid can be further enhanced, and the consequence of feature loss caused by pooling can be alleviated.

Analysis is made based on Figure 4. First, the pass through method is used to split the input feature map of the latter layer (*i* − 1) − *th* layer into four sub-blocks with the same size as the current layer (*i*) − *th* layer. They are spliced in the channel dimension in a fixed order. Then, the splicing results are reconstructed and spliced with the current layer (*i*) − *th* layer, and the 1 × 1 convolution is performed.

The input offset will cause significant changes to pooled output, as shown in Figure 5.

This shows that when the input feature graph shifts to the right by 1 feature point, the maximum pooling result will change significantly before and after the migration. For example, the input (*i*) − *th* layer is [0, 0, 1, 1, 0, 0, 1, 1]. Its average difference is divided into two sub-blocks [0, 1, 0, 1] and [0, 1, 0, 1]. The input before the offset is [1, 1, 1, 1]. What's more, the input after the offset is [0, 1, 0, 1]. Hence, the convolution kernel parameter is set to be equal to 1. Before the offset, perform 1 × 1 convolution for [0, 1, 0, 1], [0, 1, 0, 1] and [1, 1, 1, 1] to obtain [1/3, 1, 1/3, 1]; after the offset, perform 1 × 1 convolution for [0, 1, 0, 1], [0, 1, 0, 1] and [0, 1, 0, 1] to obtain [0, 1, 0, 1]. It can be seen that the convolution fusion results corresponding before and after the offset are closer. If the convolution core parameters are trained and optimized, the difference between the convolution fusion results before and after the offset can be further reduced. The convolution fusion method proposed in this paper can suppress the interference of pooling to the detection accuracy and achieve higher detection accuracy with fewer parameters and operations.

The RFM module is deployed on the DPFPN-Net vl architecture to construct a three-feature pyramid structure network DPFPN-Netv2.

## 3. Commodity Classification Based on Gradient Truncation Convolutional Network

On the basis of Multiway Integrated Dense Connection Convolutional Network(MWI-DenseNet), the connection blocks and transition layers are optimized to create a new GTNet, and the institutional differences are shown in Figure 6 below:

In the optimized structure, GTNet split the input feature graph *x*_0_ on the channel dimension to *x*_0_′ and *x*_0_^″^, and the ratio of the latter is the resolution ratio *β*. After that, *x*_0_^″^ was input into the MWI-Dense block [24–26]. After completing the n-layer convolution calculation, the dense combination feature graph *x*_*n*_ was finally output, which was input into the first transition layer to obtain the output value *x*_*t*_. It was used to connect to *x*_0_′ and then input it into the second transition layer to finally obtain the fusion output *x*_*c*_.

Taking the weight of convolution kernel as an example and excluding other parameters, the extraction features of MWI-DenseNet forward propagation and parameter optimization process of back propagation are analyzed. The mathematical expression of forward propagation process of the transition layer and each layer in the original dense connection block is as follows:

(1) $$\begin{array}{c} x_{1}=H_{1}\left(W_{1},x_{0}\right), \end{array}$$

(2) $$\begin{array}{c} x_{2}=H_{2}\left(W_{2},\left[x_{0},x_{1}\right]\right), \end{array}$$

(3) $$\begin{array}{c} x_{2}=H_{3}\left(W_{3},\left[x_{0},x_{1},x_{2}\right]\right). \end{array}$$

Here, *x*_*i*_ is the output characteristic graph of the ith layer, *H*_*i*_(·) represents the linear transformation of the *i*-th input, and *W*_*i*_ refers to the weight set of the convolution kernel at the *i*-th layer.

Input the combination feature graph *x*_*n*_ into the transition layer to obtain the output value *x*_*t*_ of the current stage:

(4) $$\begin{array}{c} x_{t}=H_{t}\left(W_{t},\left[x_{0},x_{1},x_{2},\ldots ,x_{n-1},x_{n}\right]\right). \end{array}$$

The update process of back propagation of each layer weight is expressed as follows:

(5) $$\begin{array}{c} W_{1}^{\prime }=f_{bp}\left(W_{1},g_{0}\right), \end{array}$$

(6) $$\begin{array}{c} W_{2}^{\prime }=f_{bp}\left(W_{2},g_{0},g_{1}\right), \end{array}$$

(7) $$\begin{array}{c} W_{3}^{\prime }=f_{bp}\left(W_{3},g_{0},g_{1},g_{2}\right), \end{array}$$

(8) $$\begin{array}{c} W_{n}^{\prime }=f_{bp}\left(W_{n},g_{0},g_{1},g_{2},\ldots ,g_{n-1}\right), \end{array}$$

where *g*_*i*_ is the gradient set of loss function about weight *W*_*i*_, *f*_*bp*_(·) is the weight optimization algorithm updated by back propagation, and *W*_*i*_′ is the weight after completing a round of update.

Weight updating algorithm of the transition layer is as follows:

(9) $$\begin{array}{c} W_{t}^{\prime }=f_{bp}\left(W_{n},g_{0},g_{1},g_{2},\ldots ,g_{n-1},g_{n}\right). \end{array}$$

If the network depth reuses shallow gradient information to update the weight, it will constrain the efficiency of network operation and affect the ability of network learning.

In the optimized structure, the forward propagation process of dense block and two-layer transition layer is shown as follows:

(10) $$\begin{array}{c} x_{n}=H_{n}\left(W_{n},\left[x_{0}^{\prime \prime },x_{1},x_{2},\ldots ,x_{n-1}\right]\right), \end{array}$$

(11) $$\begin{array}{c} x_{n}=H_{n}\left(W_{t},\left[x_{0}^{\prime \prime },x_{1},x_{2},...,x_{n-1},x_{n}\right]\right), \end{array}$$

(12) $$\begin{array}{c} x_{c}=H_{t}\left(W_{c},\left[x_{0}^{\prime },x_{t}\right]\right). \end{array}$$

The dense block and the first transition layer perform the back propagation process, which inputs *g*_0_^″^ to replace *g*_0_, and the weight back propagation process is shown as follows:

(13) $$\begin{array}{c} W_{n}^{\prime }=f_{bp}\left(W_{n},g_{0}^{\prime \prime },g_{1},g_{2},\ldots ,g_{n-1}\right), \end{array}$$

(14) $$\begin{array}{c} W_{t}^{\prime }=f_{bp}\left(W_{n},g_{0}^{\prime \prime },g_{1},g_{2},\ldots ,g_{n-1},g_{n}\right), \end{array}$$

(15) $$\begin{array}{c} W_{c}^{\prime }=f_{bp}\left(W_{c},g_{0}^{\prime },g_{t}\right). \end{array}$$

The synchronous comparison shows that the gradient information of updating *W*_*t*_′ and *W*_*t*_′ is not consistent, which indicates that the transition layer is split into two parts, and the shallow layer gradient information cannot enter the deep layer for weight update.

## 4. The Commodity Image Detection and Classification Model Constructed in This Study

The commodity image detection and classification model constructed in this paper based on the aforementioned methods is shown in Figure 7.

The process of Commodity inspection and classification is listed as follows:

  Step 1: initialize the parameter weight *W* and bias *b*.
  Step 2: first, the input conv6_1, conv6_2 and conv6_3 were carried on DPFM fusion. The output fusion feature graph was used as the input of the second DPFM. Then, the input conv6_3 and conv5_8 were combined to perform DPFM fusion again, and a 4-layer fusion feature pyramid 1 was constructed.
  Step 3: fusion feature pyramid 1 through the bottom-up fusion path to achieve RFM cycle fusion, so as to build fusion feature pyramid 2.
  Step 4: the prediction layer solves the predicted value and determines the loss situation;
  Step 5: back propagation, updates parameter weight *w* and bias *b*;
  Step 6: repeat the above steps until the set iterative termination times *T* is reached;
  Step 7: show the prediction results in the output picture, including the bounding box and the bounding box confidence.
  Step 8: combined with the detected images, the new GTNet network is used to classify the commodity images, and the classification results are output.

## 5. Experimental Verification

### 5.1. Construction of Experimental Environment

This experiment is carried out on the Ubuntu platform of Linux operating system, using TensorFlow framework and Python programming language. Training data are matched by an online enhancement method. After the completion of a round of training, different amplification methods are randomly referenced for data update, but there is no need to perform data amplification in the network test stage.

### 5.2. Network Structure and Parameters

The FPN-NET v2 backbone network structural parameters are listed in Table 1.

In each Conv layer, after convolution, it is connected with the BN layer and activation function layer (ReLU function is selected). Therefore, the convolution layer is equivalent to the combination layer of “convolution + BN + activation function.” By circularly fusing the original feature map of 6 layers with 4 DPFM, a fusion feature pyramid of 5 layers is constructed to construct FPN-Net vl. By circularly fusing feature pyramid 1 of 4 RFM, a fusion feature pyramid 2 of 5 layers is constructed to jointly build the FPN-Net v2.

### 5.3. Commodity Inspection Results

The Tensorboard tool is used to realize the visualization of network training-related indicators, and the change of Net v2 training loss value are shown in Figure 8.

It can be seen from the figure that in the process of increasing epoch, the loss value of network training slowed down, and the loss value stabilizes at 2.5, which means Net v2 training convergence.

In this experiment, the test data were divided into three categories: small ∈ (0,128 × 128], media ∈ (128 × 128,256 × 256], large ∈ (256 × 256,512 × 512]. The size of the test set was 512 × 512. The experimental results of FPN-Net vl, FPN-Net v2, RetinaNet detection algorithms are listed in Table 2.

According to the analysis of experimental results about the above table, all the test indexes of FPN-Net v2 are higher than other detection algorithms. If the AP_0.5_ is selected as the evaluation index, it can be found that the AP_0.5_ of FPN-Net v2 is 88.61. However, because the FPN-Net vl is equipped with fusion mechanism, the detection accuracy of small size objects is improved. On this basis, the FPN-net v2 uses the recombination fusion module to further improve the detection accuracy of small size objects.

The parameters and operation market of the aforementioned models are listed in Table 3.

Where the different circles correspond to different models and the radius of the circle is proportional to model AP_0.5_. The larger the area of the circle and the closer the center of the circle to the upper left corner is, the faster the speed for the model to achieve higher detection accuracy is. On the whole, the circle corresponding to FPN-Net vl model is closer to the upper left corner. Comparing the same ideas, the circle corresponding to the FPN-Net v2 model is closer to the upper left corner than the FPN-Net vl model, which shows that the FPN-Net v2 model has advantages in terms of detection accuracy and inference speed.

### 5.4. Commodity Classification Results

The Tensorboard is used to realize the visualization of various indicators required by network training, and the split ratio *β* = 0.5 is set. The loss of network training is shown in Figure 9.

To analyze Figure 9, it can be seen that after the network training beginning, the epoch value is gradually increased, and the network loss is overall in a decreasing trend. However, the decreasing speed is slowing down, and it finally stabilizes around Loss = 0.9. At this point, the network training process has completed convergence.

The accuracy curve of network training verification set is shown in Figure 10.

Here, after several rounds of network training, the classification accuracy of the network for verification sets keeps increasing and finally stabilizes around 99%, which has reached the requirement. It indicates that the network has a good learning fit for training data.

To test the actual accuracy of the network, the labeled target area is cut out from the original image, and the pixel value of “0” is expanded to 224 × 224. Hence, the classification test data set was obtained. Considering that the original labeled area sizes of classified images are different, to understand the impact of different size targets on network performance, the sample images in the test data set are divided into three categories: small∊(0,128 × 128), media∊(128 × 128, 256 × 256), and large∊(256 × 256, 512 × 512).

The partial classification test results of GTNet for classification test data sets are listed in Figure 11.

Here, when the split ratio *β* = 0.30, the GTNet has the highest classification accuracy, and the classification accuracy of GTNet is higher than that of MWI-DenseNet for all kinds of test sets. It means that the deep gradient flow cut-off mechanism has the application advantages, and it can improve the classification accuracy of the network.

When the split ratio *β* = 0.50, the input feature graph is half-input into the connection block and the transition layer. At this time, the classification accuracy of GTNet for the four types of test sets is still higher than that of MWI-DenseNet, and the overall computation is reduced.

When the split ratio *β* = 0.70, more input feature maps are connected to the transition layer through identity mapping, which directly affects the test accuracy of GTNet. However, at the same time, the computation is greatly reduced, and the whole reasoning process is relatively fast.

In this paper, the Billion floating point operations (BFLOPs) are used to evaluate the network computation. The GTNet network test results are listed in Figure 12 below:

It can be seen that under the conditions of different splitting ratio, the computations of GTNet are less than that of MWI-DenseNet. With the change of splitting ratio, the computations and accuracy rate of GTNet will also change.

When the split ratio *β* = 0.30, compared with MWI-DenseNet, the computation of GTNet was reduced by 3.2%. When the split ratio *β* = 0.5, the computations of GTNet are 12.7% less than that of MWI-DenseNet. When the split ratio *β* = 0.70, only 30% of the feature graph is input to the connection block. Hence, the computations of GTNet are greatly reduced, which is 20.1% lower than that of MWI-DenseNet. It is also the lowest among all the schemes.

The horizontal coordinate represents the calculation amount, and the vertical coordinate represents the accuracy, so the coordinate system is established, as shown in Figure 13.

Obviously, the radius of the circle is proportional to the accuracy of the model. The larger the area of the circle and the closer the center of the circle to the upper left corner is, the fewer parameters required in the model reasoning process is. It means that the higher detection accuracy can be achieved. Therefore, under any condition of the split ratio *β*, the comprehensive performance of GTNet is better than that of MWI-DenseNet. Namely, the GTNet has comparative advantages in calculation amount, parameters, and accuracy.

Here, the commodity images to be identified are first input into FPN-Net v2 model to obtain the commodity detection result output1. The target boundary box is marked in the output image, making the target area cut out. The size of the target area is expanded to 224 × 224. The new product target image is input into GTNet(*β* = 0.30) model. Thus, the product classification result output2 is obtained. The product boundary box and product category are identified in the output image, as shown in Figure 14.

## 6. Conclusion

It can be seen from the research that the key problem in the commodity detection and classification of is how to improve the structure of convolutional neural network. The accuracy of commodity detection and classification can be improved by constantly optimizing the structural parameters. However, the practice of this study also shows that the accuracy can reach more than 85% when the above method detects the commodities of different sizes, especially the small target commodities. Meanwhile, the amount of computation is smaller than other algorithms. However, there are limitations to the above research, that is, there is no preprocessing of image features.

## Figures and Tables

**Figure 1:** DPFM + RFM fusion feature pyramid convolution network structure.

**Figure 2:** Feature fusion module.

**Figure 3:** DPFM + RFM fusion feature pyramid detection network.

**Figure 4:** Recombination fusion module.

**Figure 5:** Schematic diagram of input offset changing pooled output.

**Figure 6:** GTNet and MWI-DenseNet connect blocks with transition layer structures. (a) Structure of MWI-DenseNet connection block and transition layer. (b) Structure of GTNet connection block and transition layer.

**Figure 7:** Block diagram of commodity identification algorithm.

**Figure 8:** Loss value curve of network training process.

**Figure 9:** Loss value curve of network training process.

**Figure 10:** Network training process verification set accuracy curve.

**Figure 11:** GTNet network test results (unit:%).

**Figure 12:** GTNet network test results (unit:%).

**Figure 13:** Scatter diagram of each model's accuracy and calculation amount.

**Figure 14:** Image recognition results.

**Table 1:** FPN-NET v2 backbone network structural parameters.

Group	Block	Layer	Output

	Input		512 × 512 × 3
Conv1_x	Initializer block		128 × 128 × 32
conv2_x	MWI-dense block 1	Layer × 6	64 × 64 × 64
	Transition layer	1 × 1 conv; pooling; SE module	
conv3_x	MWI-dense block 2	Layer × 12	32 × 32 × 256
	Transition layer	1 × 1 conv; pooling; SE module	
con\4_x	MWl-dense block 3	layer × 24	I6 × 16 × 256
	Transition layer	1 × 1 conv; pooling; SE module	
conv5_x	MWI-dense block 4	layer × 8	8 × 8 × 256
	Transition layer	1 × 1 conv; SE module	
conv6_x	conv6_l	conv3 × 3,*s* = 2	4 × 4 × 512
	conv6_2	couv3 × 3,*s* = 2	2 × 2 × 512
	conv6_2	conv3 × 3,*s* = 2	1 × 1 × 512

**Table 2:** Test results of FPN-Net and various test models (%).

Model	Backbone	AP_0.5_	AP_0.7_	AP_0.9_

RetinaNet-50	RetinaNet	86.05	65.37	45.02
FPN-Net vl	MWI-DenseNet	86.96	70.15	45.27
FPN-Net v2	MWI-DenseNet	88.61	72.03	45.92

**Table 3:** AP_0.5_ (%), number of parameters and reasoning time (ms) for each model.

Model	Number of parameters	AP_0.5_	Inference time (ms)

RetinaNet-50	30.4 M	86.05	90
DPFPN-Netv1	25.7 M	86.96	51
DPFPN-Netv2	25.8 M	88.61	52

## Data Availability

The experimental data are available upon request.
